RETRACTED

# Machine Learning Technique to Detect and Classify Mental Illness on Social Media Using Lexicon-Based Recommender System

**DOI:** 10.1155/2022/5906797

**Published:** 2022-02-26

**Authors:** B. Sumathy, Anand Kumar, D. Sungeetha, Arshad Hashmi, Ankur Saxena, Piyush Kumar Shukla, Stephen Jeswinde Nuagah

**Affiliations:** ^1^Department of Instrumentation and Control Engineering, Sri Sairam Engineering College, Chennai, India; ^2^School of Computer Science and Applications, REVA University, Bangalore, India; ^3^Department Electronics and Communication Engineering, Saveetha School of Engineering, SIMATS, Chennai, Tamil Nadu, India; ^4^Department of Information Systems, Faculty of Computing and Information Technology in Rabigh (FCITR), King Abdulaziz University, Jeddah, Saudi Arabia; ^5^Indus Institute of Information & Communication Technology, Indus University, Ahmedabad, Gujarat, India; ^6^Computer Science & Engineering Department, University Institute of Technology, Rajiv Gandhi Proudyogiki Vishwavidyalaya, (Technological University of Madhya Pradesh), Bhopal 462033, India; ^7^Department of Electrical Engineering, Tamale Technical University, Tamale, Ghana

## Abstract

The emergence of social media has allowed people to express their feelings on products, services, films, and so on. The feeling is the user's view or attitude towards any topic, object, event, or service. Overall, feelings have always influenced people's decision-making. In recent years, emotions have been analyzed intensively in natural language, but many problems still have to be watched. One of the most important problems is the lack of precise classification resources. Most of the research into feeling gradation is concerned with the issue of polarity grading, although, in many practical applications, this relatively grounded feeling measure is insufficient. Design methods are therefore essential, which can accurately classify feelings into a natural language. The principal goal of the research is to develop an overflow of grammatical rules-based classification of Indian language tweets. In this work, three main challenges are identified to classify feelings in Indian language tweets and possible methods for tackling such issues. Firstly, it has been found that the informal nature of tweets is crucial for the classification of feelings. Based on the tweets, the mental illness of the person has been classified. Therefore, to categorize Indian language tweets, a combination of grammar rules based on adjectives and negations is proposed. Secondly, people often express their feelings with slang words, abbreviations, and mixed words. A technique called field tags is used to include nongrammatical arguments such as slang words and diverse words. Thirdly, if a tweet is more complex, the morphological richness of the Indian language results in a loss of performance. The grammar rules are embedded in N-gram techniques and machine learning methods. These methods are grouped into three approaches, which functionally predict Indian language tweets with syntactic words.

RETRACTED

## 1. Introduction

The increase in social media and users' numbers has made it possible to express one's opinion in natural language. Social media feeling analysis in recent years has been an active field of research. A model needs to identify different social media [1] users' dimensions of feelings to analyze this natural language management system. The detailed review of sentimental [2] models of analysis shows that the study can assist the user to classify the operator's feelings on a theme. Analysis of the emotions is used to find user feelings or opinions. An individual has his own space in social media, such as Twitter, to post an idea or topic or comment on a service. The user review shows that various models of sentiment analysis in natural languages have been developed, film reviews, product reviews, political reviews, and so forth, for feelings analysis. In Twitter, research is being conducted extensively to predict the public mood used in different fields and applications. The classification of sentiment, in general, is divided into 3 types: (i) approach to master learning, (ii) a hybrid teaching approach, and (iii) analysis of sentiment requiring a detailed analysis of techniques of natural language processing, so that training datasets for machine learning and feeling lexical data can be provided for statistical or semantic methods. This study is aimed at developing the user's sensation framework for Tamil tweets. Nonnative English speakers have been highly influenced by social media such as Twitter. There are different discourse challenges for nonnative English speakers when expressing an opinion on social media. The first challenge is to develop grammar rules for classifying feelings in Tamil tweets. The second problem is that there are insufficient resources, such as dataset and feeling lexicons. The last question is to improve slang words' performance, words transliterated in various languages and fields.

It is not very easy to precisely identify user feelings from domain to domain by this domain-dependent word. Based on these hypotheses, the research will be validated.

  Hypoproposed work 1: concerns about the inclusion of syntactic methods for the necessary results for further improvement.
  Hypoproposed work 2: the rule-based grammar approach can better represent tweet feelings.
  Hypoproposed work 3: grammar rules combined with the supervised master method of learning improve results.

RETRACTED

The following general and specific objectives have been identified to address the challenges linked to the above-mentioned research problems. Techniques are developed for the classification of Tamil tweets based on grammar rules. Besides, this paper proposes the principal component of the sentiment analysis scheme. The proposed regulations on language grammar for Tamil tweets' classification are a characteristic feature by which user feelings are identified, and tweets are grouped into a set of categories. The work proposed contributes to new grammar rule-based algorithms for the Tamil tweets. These grammatical rules are relevant to user tweet categorization. The main tasks are to reach the elemental powers in classifying tweets and are also generic enough for various fields and systems. The Tamil tweets classification is further developed by incorporating syntactic measures such as domain-specific and tweet tags. The main idea is to add domain words to the user phrase to improve the performance of classification. The work focuses on the variety of gender instead of polarity-based systems. There are few types of research on the sort of user texts by genre. The adjective grammar shows the way for sentiment analysis in a language like Tamil. Although the Tamil language has complicated instructions, this proposed work invokes only negative guidelines and procedural regulations to categorize tweets into dissimilar categories. The planned grammar rules focus on adjectives, negatives, and connection words only to deal with ungrammatical tweet structure. This paper has proposed a new model combining syntactic, semantic, and supervised methods of learning. In general, the work is more accurate than the existing systems—also, the model is more exposed to different areas and comparison of results.

The purpose of this effort is to propose a new method for Twitter sentiment analysis, which is divided into two stages. First and foremost, there is the tweet jargon, which includes emoticons and other symbols. The emoticons are converted to plain text by using processes that are independent of the language being used. Alternatively, it is readily adaptable to multiple languages. Second, the generated tweets are categorized based on their subject matter. BERT is a language model with the advantage of being pretrained on plain text rather than tweets. The models are based on plain text and are readily accessible in various languages, reducing the need for time and resources to create them. The following advantages are accessible: (1) models may be trained directly on tweets from scratch and (2) available plain text corpora are bigger than tweets only corpora, allowing for higher performance. A case study detailing how the technology was put to use the approach for Italian is provided, along with a comparison to various Italian options that are currently available. Findings demonstrate the efficiency of the technique and suggest that, as a result of its basic foundation from a theoretical perspective, from a methodological standpoint, it has the potential to be useful for other languages as well.

RETRACTED

## 2. Literature Survey

The terms exchange of opinion mining and sentimentality examination are used by most of the current approaches. Opinion mining is defined as identifying the emotional tone underlying a piece of text using natural language processing (NLP) [3].

(1) $$\begin{array}{c} Mining\;based\;on\;Option=\;\left(u,t,i,J\right). \end{array}$$

In the above formula, “*u*” is the view objective, “*t*” is the opinion on the goal, “*i*” is the view owner, and “*J*” is the period once the idea was published. It is essential to note from the above definition that feeling mining belongs to the opinion mining sector. Sentiment mining may be of a binary type or theme detection. The term sentiment analysis (SA) is used as the term for classification tasks in this proposed work. A concept of feelings analysis was first introduced in [4]. In sentiment examination, there are three main classification methods: machine learning methods, lexical methods, and hybrid methods [5, 6]. The applied classifier of feelings depends on the data annotated. Usually, these training data are derived from function words to categorize novel information. The results of the classification machine are based on methods of functional selection. Most of the trainings already conducted focus on machine learning. Despite the numerous machine learning methods used in most of the research studies, the supporting vector machine and the Naïve Bayes classifications are standard. Therefore, the current works related to SVM and NB classifiers are reviewed in the following sections and followed by lexical sentimental analysis procedures.

### 2.1. Emotion Analysis Using Machine Learning Algorithm

When the choice of feature words or courses is an essential part of using classifiers for sentiment analyses, appropriate plan of contextual features can provide more information and reduce noise opportunities. To do so, various sources of characteristic manufacturing are frequently employed [7]. The SVM is the best method for machine learning [8] to combine several domain model knowledge characteristics, syntactic reliance, previously annotated sentences, and adjectives with standard text characteristics for a performance of 86.0%.

RETRACTED

The method of classification of polarity through machine learning algorithms was proposed in most of the reviews [8, 9]. In most of the research projects, SVM is clear to the literature [4, 10, 11] because they are robust and efficient in the analytic sentiment of highly dimensioned information. The authors of [12] considered a new algorithm to find no more than 25 video and audio genre classifications. The videos with these features are classified by SVM. The authors did not take into consideration the high dimension of genre classification.

### 2.2. Mental Illness Detection Using Lexicon‐Based System

The development of lexicon or SentiWordNet is an essential work in the lexical way to describe the “structure that holds information about words and synonyms or related meanings.” The total user sentence or text polarity is then calculated with this lexicon or WordNet with an A-weighted number of all lexical components [13, 14]. Lexicons are built using polar or emotional words. Furthermore, these opposite terms are divided into two or probably three groups, based on their divergence to construct the lexicon (positive, negative, and neutral). For lexical sentimental analysis, lexical resources and knowledge are required in a particular field. The feelings of a given text or review are calculated using the lexicon based word or phrase polarity. Unigrams or N-grams are used for training classifiers in most of the machine learning algorithms [15]. However, unigrams are used in lexicons to assign polarity; therefore, the total value of the complete text polarity is calculated as a unigram. The hybrid approach finally combines both machine learning based processes and lexicon based procedures. Moreover, a method known as a linguistic rule is usually associated with a classification of lexical sentiment [15, 16]. Some research related to hybrid approaches works specifically in a variety. To identify the hybrid method, syntactic features such as word expressions and denials, as well as the structure of the original document, are used [17]. Parts of speech (POS) are methods of identifying grammatical categories of words used in the linguistic based approach. Various POS patterns or targets may be used as functions for the sentence. POS tags are combined of substances, adjectives, or verbs. These tags can then be used to specify a specific polarity or feeling topic. Natural languages other than English have been widely used recently on social media platforms, such as Twitter and Facebook. Analysis of emotions in foreign languages has grown since a few research projects have been underway to create language resources [18, 19]; for example, in Chinese, Arabic, Hindi, and Tamil, SentiWordNet, which does not exist in English, is the most common resource. However, there is still a lack of resources for sentiment analysis tasks in many natural languages. Still, in sentimental analysis, English is the most widely used language because well-defined resources, such as lexicons, corpus, and dictionaries, are present. In particular, Tamil was used more frequently on Twitter. Researchers must face new challenges to build resources like lexicons or SentiWordNet and natural languages corpus and dictionaries. As a result, there are specific resources available for these languages because research in this area is still lacking. Many linguists and researchers are now developing natural language resources. The use of the NLTK can be taken into consideration to support the SA process. It helps to understand the natural language characteristics such as Tamil and can contribute to a more accurate SA performance. While the use of NLTK is problematic, this gives a new challenge before the SA process to incorporate NLP. A few NLP tools for SA's natural languages task have recently been developed. The literature reveals the availability of various methods of machine learning for the analysis of feelings. Also, all current investigations on sentiment examination put emphasis on the organization of divergence. As for Tamil tweets, a lack of resources is the main problem in this area. To categorize the sentimentality of Tamil movie tweets, a semantic method can be practical. Three key subjects are finally examined to improve the classification of emotion in Tamil tweets: first, the method for field tags, second, the use of grammar rules by film reviews using syntactic and semantic models, and, third, the machine knowledge methods. A new grammar procedure for the proposed work predicts the Tamil genre class tweet.

RETRACTED

## 3. The Methodology of Proposed Framework

The general framework for the Tamil tweet sentiment analyses using various algorithms is explained. The design of the systems underpinning the work is first described, and then every phase of the plan related to this work is presented.  Section 3 provides a note on the structure and justification for the creation of the Tamil language. A short description of the film's genres follows/product review classifications and accuracy metrics.  Figure 1 shows how the Tamil tweets classify their sentiment.

### 3.1. Proposed Architecture of Proposed Model

Four steps of user tweets' feelings in Tamil movies are taken for identification. The first step is to collect and prepare tokenizers for all user tweets. The next process is to detect parts of voice tags with tokenized keywords. Finally, the tokenized content procedures will be used to identify the genre category using the natural language toolkit.

Figure 2 shows the general procedure included in this framework for sentimentality analyses.

#### 3.1.1. Input Data Collection

The primary stage is to gather the data needed for classification—sentiment analysis. There are in the area of sentimental analysis different well-established datasets available in English and the related domain. For natural languages other than English, only limited datasets for feeling analysis are available. In this research, all datasets are extracted from Twitter using the hashtag (#) and then the movie/product's name using Twitter's API. However, there is no predefined dataset for Tamil films; an unlabelled dataset for experimental analysis is a significant task.

The last week in July 2016 includes all of the Tamil film tweets used in this proposed work. 100 Tamil films and product tweets were collected (mobile phone). Initially, the idea was to create a film dataset only but only for the sensation framework to prove that two datasets are made independent of the domain. The body contains 7,346 tweets from Twitter which have been collected and used for all purposes.

#### 3.1.2. Preprocessing Task

The next step is the pretreatment of tweets. To remove conflicting, imperfect, and luminous information, the preprocessing of data is done. To perform all data mining functionality, data needs to be preprocessed. The first job is to delete URLs. Usually, the Uniform Resource Locator does not help in informal words to assess the feeling. For example, take the phrase “I logged on https://www.amazon.in as the film is boring.” This phrase is harmful because it is wrong and can become neutral of the amazon text's occurrence. A technique for removing the Uniform Resource Locator is used to avoid such errors. The following task is to remove retweets. Retweeting is the process of copying a tweet and posting it to a second user. This is usually if a user likes another user's tweets. Retweets are frequently abbreviated as “RT.” These retweets are redundant data to remove all retweets.

#### 3.1.3. Tokenization Process

Tokenization is a way of dividing words into different words or tokens into user tweets. A phrase, word, or symbol might be a token. The tweet phrases are tokened into a series of words that can be analyzed with white spaces to remove any specific character or punctuation marks such as # and @. The various Documentary Dictionaries are called token sets produced by combining the full text of a collection.

RETRACTED

#### 3.1.4. Sentiment Analysis Models

Supporting vector machines are commonly used to detect sentiment topics on a document level, unchecked approaches like Naïve Bayes [20]. But more advanced models, such as the linguistic rules, are required to categorize the (polarity) opinions and sensations of informal text (gender). The suggested sentiment framework is divided into three functionality-based models.  Figure 3 shows two types of feelings investigation.

### 3.2. Tools

Software access to Twitter is needed to create a tweets corpus. The Twitter REST API is used in this research to access corpus user tweets. This API also provides developers with access to all public tweets and their associated metadata to search for and download streams. However, access to data from the Twitter API is restricted. Authentication methods (OAuth) are used for user prevention misconduct. Various programmers can also use it to understand the use of the API. To access all tweets in real time, Twitter “Firehose” is the only way. Access to the Twitter “Firehose” generally comes from third-party (GNIP and DataSift) managers, although it is not free of charge. The costs of subscription for individual scientists working in sentiment analysis are very high. The streaming API can nevertheless be used to access tweets in real time with a particular number of Twitter data requests. For sentimental analysis, the Tweepy Python API is employed to collect Twitter information. If a user wants to use Twitter API directly, the TWIP connection is relatively complex. It enables user-friendly search and download functions. Usually, the relationship with the routine is established.

#### 3.2.1. Twitter API

The NLP has developed a portion of the speech tags to classify the words according to their POS. A portion of the speech tagger helps in the analysis of the feelings for the two reasons: (1) it may be used to differentiate words that are not generally felt in POS and (2) words such as pronouns and nouns can be used with POS.

The classification task POS tag in [21] is used in this proposed work. The Python Requests framework was developed to manage HTTP requests using the POS tagger.  Figure 4 illustrates an example of a tagged tweet in that POS tagger.

The TF-IDF for document or word classification is a simple unigram model. TF-IDF works well in the classification of documents, such as news articles or reviews [22]. The literature shows, however, that TF-IDF does not classify tweets as well as long tweets and does not follow grammatical styles, and general words are seldom repeated. Tweets, however, contain valuable information for the extraction of feelings. As a basic model, TF-IDF is chosen; it gives the meaning of the word in a dataset. Set of words in tweets should correspond to the subjects and the most frequently reported words should be obtained. To classify the tweets [23] into a set of data, the top *N* TF-IDF keyword values of each film are selected. Consider a film *mi* that is linked to a set of tweets {t1,t2..... Tn}, where Tn is translation. There are several terms in each tweet which allow each film to be marked.

RETRACTED

The group of words *x*1, *x*2,....*xk* are like a tweet sequence.

(2) $$\begin{array}{c} mi=\left\{u1,u2,\ldots ,un\right\}=\left\{x1,x2,\ldots ,xk\right\}. \end{array}$$

Also, every movie can be considered as a tweet group.

Their associated tweets contain a set of words, *tf*, *mi*, and idolatrous (*wj*, *m*).

The values are calculated as follows:

(3) $$\begin{array}{c} tf\left(x_{j},n_{j}\right)=\frac{\;input\;co-occurence\;frequency\;of\;x_{j}}{n_{i}},\\ idf\left(w_{j},m\right)=\log\left(\frac{\;overall\;emotional\;tweets\;of\;the\;person\left(n\right)}{\;input\;co-occurence\;fequency\;of\;overall\;tweets\;}\right). \end{array}$$

Take a movie “Veeram” with 305 tweets as an example.

Where the word is twenty times (Rasool) and the word is 18 times.

Total dataset tweets are as follows:

(4) $$\begin{array}{c} tf_{rate\;}=\frac{20}{305}=0.0656,\\ idf_{rate\;}=\log\frac{305}{18}=1.229,\\ tfidf_{rate\;}=tf*idf=0.0806. \end{array}$$

Similarly, the TF-IDF is calculated and the important keywords can be identified with the score for all the genres that correspond to the domain. The synonyms of the selected keywords are also mapped with the Tamil dictionary to reduce dimensionalities and improve the performance of the category and word model [24].

## 4. Algorithm for TF-IDF

The sentiment categorizer model is used after data collection and preprocessing to achieve the following in the baseline model:

1. Divide all tweets into keywords or tokens.
2. Identify the occurrence and related words in the tweet for each keyword.
3. For every keyword selected from a user's tweet, compute the TF-IDF score.
4. Multiply TF-IDF with SentiWordNet's Tamil score.
5. Set all user tweets with mean precision in the overall sentiment scores.
6. Assign a film by Step 5 to genre and polarity.

The image of user tweets [24] for the sentiment classes is shown in Figure 5 (Veeram). The result shows the proportion of polarity and gender tweets. Although Action and Trade point were verified by domain professionals, the film genre class has shown that it is categorized into a comedy genre (23, 60%) and love (23.88, 21%). The TF-IDF approach relies on a unigram or perfect keyword and categorizes a tweet only when the keyword is available. The TF-IDF model also does not take into account the user tweet context.

RETRACTED

### 4.1. Algorithm for Genre Classification

The syntax parser determines a tweet's overall polarity and gives this score a perception categorizer model to determine a tweet's type class.  Figure 6 shows the algorithm used to classify sentiments.

The tweets are identified with the syntax parser and POS taggers result using the above algorithm in the Categorizer Sensitivity Model [25]. The tweet is classified in an adjective way into the closely related class when the polarity of a tweet is positive. Extraction from parser-based negation produces a greater accuracy than syntax models of 47.32 percent. The rules on negation are designed to improve the analysis of feelings. The findings show that the model of grammatical negation dependence has a higher level of efficiency in sentiment analysis compared with frequency and other syntactic models [26]. The results show that the variety of evolving user-generated text needs to be dealt with throughout the grammar rule approach.

### 4.2. Adjective‐Based Grammar Rules for Semantic Model

This work is hypothesized by the adjectives as the principal semantic structure for the classification of film genres. Most of the Tamil grammarians speak only of substances and verbs. It is said that adjectives are not considered as separate categories in Tamil by traditional grammarians or linguists. Adjectives are used for the description or quantification of a noun object. Adjectives differ in occurrence and function in different languages. In modern Tamil, adjectives are mostly written just before the substrate. A pattern of adjectives concerning Tamil film tweets is identified by this method [24]. These adjective patterns are linked directly to the specific domain posts and thus rules for finding an impression of the specific posts have been developed in this context. Adjectives are also used to express the strength of user feelings by intensifying them.

Grammar modification is as follows: temporary values {+2} in the application of rules 2 and 3 temporary scores are derived. Upon application of the rules, the initial results are not altered because the tweet has no other opinions or terms of denial. Final score is {+0.66}.

The endpoints are standardized between +1 and −1. The final result is calculated with two divided by three, for example, in this case.

(5) $$\begin{array}{c} \text{Final score}=\frac{\text{Adjective score of the input data}}{\text{Analysed words in the sentence of the system }}. \end{array}$$

The match calculation undergoes by an action point. The category match calculation: Action (+).

### 4.3. Supervised Model

The characteristics of the classifiers should be extracted for machine learning classification. Functional vectors affect the classifiers' performance [27]. Two methods of extraction, character presence and character count, are generally used specifically. Character count uses the count of frequencies (if the count of frequencies is high, the word is considered to be the word character), while the character presence uses the characteristic word's presence or absence. Although tweets are short, this work uses the function presence method for the extraction of functions. The first five (unigrams) adjectives correspond to the initial seed list for each genre [28]. The seed list synonyms and antonyms are derived from a software programme, Tamil WordNet. This process continues until all functional adjectives have been added to the functions list.  Table 1 represents the kernel adjectives.

RETRACTED

At first, 500 corpus tweets are selected manually to train the classification. Each tweet will extract the words of the function (93 adjectives in this book) from the list and other words will not be taken into account. Similarly, for instantiation of SVM classification, the NLTK library file is used. It is noticed that several tweets occur repeatedly through multiple posts of the individual user in the corpus. There are also some tweets with misleading feelings or feelings about the specific field. The performance of the classifiers will degrade if such tweets are selected as a set for training. The experiment is conducted with NLTK library files for both classifications. For both classifiers, 10-fold cross-validation is made.

Computational learning theory is behind the support vector machine (SVM) machine learning technology. SVM's main purpose is to find the most efficient classification function for categorizing the training dataset's classes. To handle linear and nonlinear classification issues like density estimation or pattern recognition, the SVM model is commonly utilized. Translate the training data into a higher dimension using nonlinear transformation, and then divide it into separate training sets using the linear method.

A kernel function *K* is replaced for the intermediate product (*X*, *Y*) in a nonlinear SVM classification model (*X*, *Y*):

(6) $$\begin{array}{c} f\left(x\right)=sign\left(\sum_{j=1}^{W}bx_{j}K\left(x_{j},x\right)+c\right). \end{array}$$

In the learning process, SVM employs a two-layer structure. It is the initial layer that selects the kernel's base *K*(*x*_*i*_, *x*), where *i* is one of 1, 2, 3, 4, 5, or 6. Layer 2 is a linear function in the feature space formed by the first layer. Making the best hyperplane in the similar feature space is the same as it was in the previous example. It is generally accepted that hyperplanes with bigger margins are more accurate than hyperplanes with smaller margins when used to categorize feature data. The shortest distance between the hyperplane and the margins on each side is taken to be the hyperplane with the greatest margin. Hyperplane for separating planes is defined by the following equation:

(7) $$\begin{array}{c} W_{-}X+c=0. \end{array}$$

Margins are determined as the support vector points. The outcome of the process is the linear combination of all support vector points, and all other data points are overlooked. It comes with the notion that the complexity is not dependent on the number of features existing in the training dataset. It makes SVM very efficient for classification problems that hold a considerable number of features as compared to the number of training examples. The only drawback with SVM is that, in case of misclassified or linearly inseparable data, no separating hyperplane can be obtained. So, the SVM translated the data into higher dimensional feature space and found a suitable hyperplane. In this work, the LS-SVM Lab toolbox has been applied to classify the speech of ID from TD children. To achieve a better classification accuracy, the two regularization parameters, (*γ*, gam) and *σ*2(*sig*2), which was the squared bandwidth of RBF kernel, have been chosen optimally.

RETRACTED

## 5. Experimental Results

An analysis tool was developed which incorporates all NLTK-based and Python-based algorithms. The tool shows automatically the feeling values of Tamil movie tweets both at the polarity level and at the genre level.  Figure 7 shows the feelings for the Veeram film.  Table 2 represents the grammar performance.

The results suggest that the general sentiment model based on the grammar rule delivers better performance compared to other syntactic models. The results also show that the precision sentimental analysis increases significantly when somaticized models in addition to normal functionality like unigrams are incorporated (TF-IDF). Compared to other feeling models, the grammar approach proposes the semantic structure of the user's phrase within the specific domain.

The semantic grammatical model provides an average accuracy of 64.72 percent better than that shown in Figure 8 for TF-IDF and other syntactic models. Sentiment model has analyzed tweets and found polarity, genre categories, and other algorithms using proposed grammar rules. Results demonstrate that the general grammar of negative rules and adjective rules is better because complex sentences are taken into consideration and semantic structures are better integrated. The proposed grammar rules address any sort of sentence in tweets to determine sentiments (simple, compound, and complex). The grammar rule-based model with an accuracy of 64.72 percent is the best feeling model. If the results of TF-IDF, tweet weight, and regulatory modeling are compared, the grammar-based algorithm could be found to be 20 percent better than other sentiment models. The results show that machine learning methods alone are not good for feelings. One of the important lessons of this is that, instead of using the grammar methods, SVM is better than the syntax model. The classifier quality is only as high as the set, so all possible instances cannot be exposed to the classifying system. Therefore, to improve machine study classifier performance, adjective and negative-based grammar rules are used as a feature for classifiers to compare machine study methods with grammar rules.  Table 3 shows the SVM classification performance in combination with grammar regulations.

RETRACTED

When the grammar rules are combined with the SVM classification, it is determined to outperform all other feelings models in combination with the grammar rules method. Between the grammar rule and learning models, the accuracy changes 7%. The result highlighted again the quality and the ambiguity of Tamil grammar in the grammar-based machine learning model. A good promise is made with grammatical rules for further development. For cross-domain assessments mobile phone reviews, the proposed sentiment framework procedures are adapted. This is because the number of tweets available on this domain is the number of movie domain choices. The aim is to verify the performance of the grammar rules algorithms and methods of machine learning regardless of domain even if the size of the product field tweets is small. The domain-independent features for the training are extracted for master classification. The words that occur in all domains are domain-independent characteristics. This function is important for transferring the semantical context from one domain to another. The grammar rules are used in this research work to extract independent domain adjectives for analysis of cross-domain feelings.  Table 4 shows the results of each of the three models of feeling.

The study shows that the algorithms work in a comparable way for different domains. This demonstrates the work's expansion into various areas.

## 6. Conclusion

The present dataset has been applied to the existing algorithms like SVM and Naïve Bayes, and results were tracked. The results show that SVM model could better classify the genre of film compared to syntactic methods. The work thus suggested that both models be combined and the results traced. While the proposed algorithms with the setup of a feeling framework are successful, it is valuable to assess their performance with the system's composition in real time. The proposed model would then be tweeted in real time as part of future work.

RETRACTED

The overall model could be changed if the work is carried out in real time. In future work, this is an important direction. If work continues, lexical resources must be developed when this research is extended to more than one area. The focus of this research has so far only been two areas (films and product), and the domain tag resources for these two areas have therefore been developed. Once the grammar models for the complex phrases are completed, the paragraphs can also extend the model. It is also essential to implement a grammar-regulative approach for handling complex and composed sentences as a cause of the error. The future will automatically focus on “generate tags” (types) from the text. The SVM, in combination with the rules of grammar, outperforms all other Tamil tweets in feeling analysis. This is an essential finding of the approach to machine learning. Two product category tweets were used, and the sentiment methods were applied to track the validity of the model in various domains. These results have been validated so that the grammatical techniques are efficient. There has been no significant improvement in outcomes when combining SVM with grammar-based techniques. The other two machine methods can also be tested in future work (Semisupervised and Unsupervised).

## Figures and Tables

**Figure 1:** Sentiment analysis framework for Tamil movie tweets.

**Figure 2:** Flow chart of proposed work.

**Figure 3:** Three types of sentiment models.

**Figure 4:** Input tagging.

**Figure 5:** Sentiment model using TF-IDF.

**Figure 6:** Algorithm for genre classification.

**Figure 7:** Results of feeling analysis by grammar rules.

**Figure 8:** Performance comparison of grammar-based semantic models with TF-IDF.

**Table 1:** Instance list of early kernel adjectives and their synesis.

Initial seed list	Synonyms	Antonyms
Action	“Fight,” “action,” “veeram”	“Peace”
Love	“Love,” “romance”	“Sogam”
Commercial	“Vasool,” “mass,” “commercial”	“Ioss”
Comedy	“Comedy”	“Tragedy”
Family	“Sentiment,” “family,” “feeling”	“Aabasam”

**Table 2:** Tamil SA grammar performance.

Movie	Method	Accuracy
Veeram	TF-IDF ranking	27.13
	TF-IDF + DST	36.42
	Tweet weight	40.26
	Negation rule	47.32
	Adjective rule	60.84

**Table 3:** Performance of SVM classifier with grammar rules.

Movie	Method	Accuracy
Veeram	TF-IDF ranking	27.13
	Domain-specific tags	36.42
	Tweet weight	40.26
	Negation rule	47.32
	Grammar rule	60.84
	SVM + grammar rules	65.73

RETRACTED

**Table 4:** Performance analysis for product domain.

Corpus	Method	Accuracy
“Mobile phone”	TF-IDF ranking	29.35
	Domain-specific tags	30.98
	Tweet weight	45.18
	Negation rule	59.97
	Grammar rule	66.82
	N-gram model	65.23
	Naïve Bayes	47.94
	SVM	58.96
	SVM + grammar rules	69.32

## Data Availability

The data that support the findings of this study are available upon request from the corresponding author.
